RETRACTED

# Characteristics of cognitive function in patients with cerebellar infarction and its association with lesion location

**DOI:** 10.3389/fnagi.2022.965022

**Published:** 2022-10-04

**Authors:** Qi Liu, Chang Liu, Yumei Zhang

**Affiliations:** ^1^Department of Neurology, Beijing Tiantan Hospital, Capital Medical University, Beijing, China; ^2^China National Clinical Research Center for Neurological Diseases, Beijing Tiantan Hospital, Capital Medical University, Beijing, China; ^3^Department of Rehabilitation, Beijing Tiantan Hospital, Capital Medical University, Beijing, China

**Keywords:** cerebellar infarction, post-stroke cognitive impairment, cerebellar lobule, functional lateralization, functional topography

## Abstract

**Objective:** This study aimed to explore the characteristics of cognitive function in patients with cerebellar infarction and its association with lesion location.

**Methods:** Forty-five patients with isolated cerebellar infarction were collected in the Department of Neurology, Beijing Tiantan Hospital. Thirty healthy controls were recruited matched by age and education. Global cognitive function was evaluated by using Addenbrooke’s Cognitive Examination version III (ACE-III). An extensive neuropsychological assessment battery was also tested to evaluate the characteristics of each cognitive domain. 3D slicer software was used to draw the lesion, and evaluate the lesions’ volume, side, and location. Group analysis was used to compare the differences in cognitive performance between patients and healthy controls, and patients with left and right cerebellar hemisphere infarction. Spearman analysis was used to explore the correlation between cognitive function and lesion volume. We also subdivided each patient’s lesions according to the cerebellar atlas to identify the specific cerebellar location related to cognitive decline.

**Results:** Patients with cerebellar infarction had a lower ACE-III score compared with the healthy group (87.9 ± 6.2 vs. 93.7 ± 2.9, *p* < 0.001), and 22 (48.9%) patients were diagnosed with cognitive impairment. The *z*-transformed score of attention and executive function in the patients’ group was −0.9 ± 1.4 and −0.8 ± 1.0 respectively, with 19 (43.2%) and 23 (56.4%) patients impaired. Compared with healthy controls, the relative risk ratio with 95% confidence interval (CI) for impairment in attention and executive function were 3.24 (1.22–8.57) and 3.39 (1.45–7.89). However, only 10 (22.1%) patients showed impairment in more than two cognitive domains. Compared with the left lesion group, patients with right cerebellar infarction showed significantly impaired executive function (−1.1 ± 0.3 vs. −0.5 ± 0.2, *p* = 0.01). And the cerebellar posterior lobe regions, especially lobules VI, VIII, and IX, were explored to have lower cognitive performance. Furthermore, lesion volume was identified to be associated with the ACE-III score (*r* = −0.37, *p* = 0.04).

RETRACTED

**Conclusion:** We identified that cerebellar involvement in cognition, especially in attention processing and executive function. Cerebellar right-sided lateralization of cognition and functional topography were also revealed in the current study.

## Introduction

The cerebellum’s role in cognition has previously been reported, in addition to its established relationship with motor control (Buckner, 2013). Cerebellar diseases can cause disturbance in executive function, damage to language processing, visuospatial dysfunctions, as well as emotional abnormalities, which have been defined as Cerebellar Cognitive Affective Syndrome (CCAS; Schmahmann and Sherman, 1998). Furthermore, functional lateralization and fine topography have been shown in the cerebellum (Paulus et al., 2004; Richter et al., 2007; Schmahmann et al., 2009; Stoodley et al., 2016). Previous neuropsychological studies found that patients with right cerebellar damage had worse cognitive performance compared with a left lesion (Shin et al., 2017; Chirino-Pérez et al., 2021). And a motor-cognitive dichotomy has been widely recognized: motor function is influenced by an anterior lobe lesion, whereas performance on cognitive tasks is more affected by lesions in the cerebellar posterior lobe regions (Paulus et al., 2004; Richter et al., 2007; Schmahmann et al., 2009; Stoodley et al., 2016).

Cerebellar stroke, in which the lesion is confined to the cerebellum and not complicated by cerebral abnormities such as atrophy or hydrocephalus, is an appropriate clinical model for researching the cerebellum’s function in the cognitive process (Ng et al., 2007). In addition, the distribution of cerebellar infarction lesions differed by vascular territory, which was deemed appropriate for studying cerebellar cognitive topography. Focusing on patients with cerebellar infarction, our study aimed to explore the characteristics of cognitive function in focal cerebellar disorders and its association with lesion location.

## Methods

### Participants

A total of 45 patients with cerebellar infarction were recruited in the Department of Neurology, Beijing Tiantan Hospital from June 2020 to December 2021. The inclusion criteria included: (1) age from 18 to 80 years old; (2) with 6 and more years of education level; (3) the first onset of cerebellar infarction; (4) admitted within 14 days of stroke onset. Exclusion criteria included: (1) pre-existing neurological/psychiatric disease; (2) chronic alcohol or drug abuse; (3) metabolic disorders, nutritional deficiencies, and infectious diseases which may influence cognitive function (Supplementary Figure 1). In addition, we also included 30 age- and education-matched healthy control participants.

RETRACTED

All participants gave written informed consent to the procedure, which had been approved by the ethics committee of Beijing Tiantan Hospital.

### Demographics characteristics and neurological examination

Demographics and clinical information were collected for each participant. Demographic information included age, sex, and educational level. Clinical information included onset duration and infarction volume. We also evaluated the motor functions of patients: the International Cooperative Ataxia Rating Scale (ICARS) was used to assess the severity of ataxia and the Brunel balance assessment (BBA) was used to assess balance dysfunction (Trouillas et al., 1997; Tyson and DeSouza, 2004). Furthermore, the self-rating anxiety scale (SAS) and the self-rating depression scale (SDS) were used to assess the possible presence of anxiety and depressive states respectively (Zung, 1965, 1971).

### Assessment of cognitive function

Patients performed the Chinese version of the Addenbrooke’s Cognitive Examination III (ACE-III) to evaluate global cognitive function. The ACE-III was designed to assess the five cognitive domains: attention, memory, verbal fluency, language, and visuospatial abilities, and its scores range from 0 to 100 points. Cognitive impairment was defined as an ACE-III score <87, which has been verified in the Chinese population (Li et al., 2019).

In addition, a battery of neuropsychological assessments was applied to further examine the main cognitive domains using the following neuropsychological assessments. Attention was assessed with Trail Making Test (TMT) A (Tombaugh, 2004) and Forward Digit Span (Wechsler, 1997). Working memory was assessed with Reversed Digit Span (Wechsler, 1998). The visuospatial function was assessed with the copy scores of the Rey Complex Figure (RCF) test (Rey, 1941). Language processing was assessed with Boston Naming Test (Kaplan et al., 2001). Episodic memory was assessed with RCF Recall (Rey, 1941) and Rey Auditory Verbal Learning Test (RAVLT; Rey, 1958). Executive function was assessed with Trail Making tests A and B (Tombaugh, 2004), phonemic and semantic (animals) verbal fluency (Spreen and Strauss, 1998; Tombaugh et al., 1999), and the Stroop test (Stroop, 1935).

### Neuroimaging acquisition and preprocessing

All participants underwent MRI on a 3T MR scanner (SIGNA Premier; GE Healthcare, Milwaukee, WI, USA) with the 48-channel head coil. T1-weighted sequences and T2-fluid attenuated inversion recovery (FLAIR) sequences were acquired. Image acquisition was performed by a trained professional who was unaware of the patients’ clinical information.

RETRACTED

Preprocessing of all images was implemented on MATLAB2021b^1^, using the Spatially Unbiased Infratentorial Template (SUIT) in SPM12^2^ (Diedrichsen et al., 2009). For each patient, cerebellar lesion areas were clearly delineated on the T2-FLAIR MRI sequence and their volume was automatically measured on 3Dslicer software^3^. Then, each patient’s lesion was spatial normalized using the normalization procedure’s deformation parameters on MATLAB. Lesions were overlain on the coronal T1-weighted template designed by Diedrichsen et al. (2009). The impaired cerebellar lobules of each patient were also evaluated using the 3D MRI atlas of the human cerebellum, determining from the MRI coordinates of the lesion images (Diedrichsen et al., 2009).

### Statistical analysis

Continuous variables were presented as mean ± standard deviation (SD) and categorical variables as frequency (percentage). Comparisons between two groups were performed using independent sample t-tests and the Mann-Whitney U tests for continuous variables, and the Chi-squared tests for categorical variables. To calculate the effect size of the differences observed between cognitive groups we used Hedge’s g coefficient, with *d* < 0.2 considered a very small effect size, *d* > 0.2 a small effect size, *d* > 0.5 a medium effect size, and *d* > 0.8 a large effect size (Hedges and Olkin, 2016). For comparison between multiple groups, one-way ANOVA and LSD tests were used.

Furthermore, raw neuropsychological scores were converted into z scores to enable comparisons across measures according to the following formula: *z*−score = (patient raw score − healthy group mean)/healthy group SD (Goff and Ackerman, 1992). For cognitive domains with multiple scores, mean (composite) values were calculated when applicable. And *z*-score of each cognitive domain for different cerebellar lobule was also evaluated. Impaired cognitive domain was defined as one or more SD below healthy group means, while severe deficits in cognitive domains were defined as a result below the mean—2SD. However, as previous studies mentioned, for the differences between an individual’s scores, a percentage of the healthy population also can exhibit one or more abnormally low test scores (Crawford et al., 2007). For tackling such problems, relative risk ratios (RR) for each impaired cognitive domain between healthy controls and cerebellar infarction patients were performed.

*P* value < 0.05 was considered to be statistically significant (2-sided). Analyses were performed using SPSS version 26.0 (IBM, Armonk, NY, United States).

RETRACTED

## Results

### Demographic and clinical characteristics

Table 1 summarized demographic and clinical characteristics. Age, sex, and education showed no significantly different between patients’ group and healthy controls. And all patients recruited in this study were right-handed. Patients had a higher SAS score when compared to healthy controls. The average onset interval day in the patients’ group was 9.0 (5.0), and the median infarction volume was 14.4 (29.6) cm^3^. The poor performance of ICARS and BBA demonstrated ataxia and balance impairment in patients with cerebellar infarction. In addition, Supplementary Table 1 showed no significant difference in age, sex, education, and infarction volume between patients with different infarct sides.

**Table 1:** Demographic characteristics of controls and cerebellar infarction patients.

	**Healthy controls**	**Cerebellar infarction patients**	***P* value**
	***n* = 30**	***n* = 45**	
Age (y)	49.9 ± 13.3	51.0 ± 12.1	0.72
Male, n (%)	26 (86.7)	41 (95.6)	0.16
Education (y)	12.2 ± 2.9	10.8 ± 2.9	0.06
Onset duration (d)	-	9.0 (5.0)	-
Infarction volume (cm^3^)	-	14.4 (29.6)
ICARS score	-	8.5 (13.0)	-
BBA score	-	10.1 ± 2.5	-
SAS score	31.8 ± 5.8	36.7 ± 6.2	0.001
SDS score	0.36 ± 0.06	0.36 ± 0.07	0.78

Continuous variables conforming to normal distribution were presented as mean  ±  standard deviation (SD), and those not conforming to normal distribution were presented as median (interquartile spacing). categorical variables were presented as frequency (percentage). Abbreviations: ICARS, International Cooperative Ataxia Rating Scale; BBA, Brunel Balance Assessment; SAS, self-rating anxiety scale; SDS, self-rating depression scale.

### Cognitive performance in patients with cerebellar infarction

Compared with a healthy group, patients with cerebellar infarction had a lower ACE-III score (87.9 ± 6.2 vs. 93.7 ± 2.9, *p* < 0.001). Twenty-two (48.9%) patients were diagnosed with cognitive impairment, while no individuals in the control group had cognitive impairment. *Z*-transformed composite scores in each cognitive domain showed that cerebellar infarction patients had significantly impaired in attention (*p* < 0.001) and executive function (*p* < 0.001; Table 2). Raw scores for each cognitive test in each group are reported in the Supplementary Table 2. The most commonly affected cognitive domains were attention, working memory and executive function, with 19 (43.2%), 23 (53.3%), and 23 (56.4%) patients affected respectively (Figure 1). However, a small proportion of healthy controls in our study also showed abnormalities in cognitive function (Supplementary Figure 2). Compared with healthy controls, the unadjusted RRs with 95% confidence interval (CI) for impairment in attention and executive function were 3.24 (1.22–8.57) and 3.39 (1.45–7.89) respectively. When education was included as a covariate, the adjusted RR with 95% CI were 4.57 (1.33–10.68) and 5.69 (1.77–8.32) for the cognitive domain of attention and executive function (Table 3).

RETRACTED

**Figure 1:** The percentage of impaired cognitive patients in each cognitive domain.

**Table 2:** *z*-Transformed cognitive scores in healthy controls and cerebellar infarction patients.

**Cognitive domains**	**Healthy controls**		**Cerebellar infarction patients**			**Effect size (Hedge’s g)**	**95% Confidence interval**
	**mean ± SD**	**Range**	**mean ± SD**	**Range**	***P* value**
Attention	−0.0 ± 0.8	−1.6–1.5	−0.9 ± 1.4	−3.5–1.8	<0.001	−0.94	(−1.45, −0.44)
Working Memory	−0.0 ± 0.9	−1.2–2.1	−0.6 ± 1.4	−5.7–2.1	0.07	−0.44	(−0.86, 0.00)
Visuospatial	0.0 ± 1.0	−3.6–0.7	−0.5 ± 2.8	−16.6–0.7	0.41	−0.24	(−0.48, 0.31)
Language	0.1 ± 0.9	−2.2–1.5	−0.4 ± 2.4	−13.7–2.1	0.54	0.18	(−0.22, 0.92)
Episodic Memory	−0.1 ± 0.8	−2.7–1.5	−0.2 ± 1.1	−4.9–1.3	0.67	−0.10	(−0.51, 0.37)
Executive Function	0.0 ± 0.5	−1.3–0.9	−0.8 ± 1.0	−3.5–0.9	<0.001	−1.00	(−1.37, −0.60)

Abbreviations: SD, Standard deviation.

**Table 3:** Relative risk ratio for each impaired cognitive domain among healthy controls and patients with cerebellar infarction.

**Cognitive domain**	**No. of outcomes (*n*, %)**		**Relative risk ratio (95% Confidence interval)**	
	**Healthy controls**	**Cerebellar infarction patients**	**Unadjusted**	**Adjusted**
Attention	4 (13.3)	19 (43.2)	3.24 (1.22–8.57)	4.57 (1.33–10.68)
Working Memory	9 (30.0)	24 (53.3)	1.78 (0.97–2.28)	2.56 (0.94–6.93)
Visuospatial	6 (20.0)	11 (25.6)	1.28 (0.53–3.08)	1.22 (0.38–3.92)
Language	7 (23.3)	6 (13.3)	0.58 (0.21–1.53)	0.39 (0.11–1.42)
Episodic Memory	4 (13.3)	7 (16.7)	1.25 (0.40–3.89)	0.87 (0.21–3.59)
Executive Function	5 (16.7)	22 (56.4)	3.39 (1.45–7.89)	5.69 (1.77–8.32)

Covariate: educational levels.

We also explored the number of impaired cognitive domain in each patient with cerebellar infarction and healthy control (Figure 2 and Supplementary Figure 2). In patients’ group, 39 (86.7%) were impaired in one or more cognitive domains, and 22 (48.9%) had two or more impaired cognitive domains. The RRs with 95% CI when compared with healthy controls were 1.73 (1.19–2.52) and 2.01 (1.03–4.28) respectively. In the current study, however, only 10 (22.1%) patients showed impairment in three or more cognitive domains.

**Figure 2:** The number of impaired cognitive domain in each patient with cerebellar infarction **(A)** and healthy control **(B)**.

RETRACTED

Furthermore, we found that the global cognitive function correlated with the severity of motor symptoms in cerebellar infarction patients (Supplementary Figure 3).

### The effect of lesion location on cognitive performance in patients with cerebellar infarction

There were no significant differences in ACE-III scores between patients with left and right cerebellar lesions (89.0 ± 5.3 vs. 86.7 ± 6.8, *p* = 0.39). While compared with the left lesion group, patients with right cerebellar infarction showed significantly impaired executive function (−1.1 ± 0.3 vs. −0.5 ± 0.2, *p* = 0.01; Table 4). Supplementary Table 3 showed right lesion group had worse performance than the left lesion group in the test of TMT, and Phonemic fluency.

**Table 4:** Comparison of *z*-transformed cognitive scores according to the lesion side after cerebellar infarction.

			**Cerebellar infarction patients**				
**Cognitive domains**	**Healthy controls *n* = 30**		**Left lesion *n* = 20**		**Right lesion *n* = 22**		***P* value**
	**mean ± SD**	**Range**	**mean ± SD**	**Range**	**mean ± SD**	**Range**
Attention	−0.0 ± 0.8	−1.6–1.5	−0.6 ± 0.3	−3.2–1.4	−0.9 ± 0.3^a^	−3.5–0.5	<0.01
Working Memory	−0.0 ± 0.9	−1.2–2.1	−0.6 ± 0.2	−2.3–1.0	−0.8 ± 0.4	−5.7–1.0	0.12
Visuospatial	0.0 ± 1.0	−3.6–0.7	0.2 ± 0.2	−1.7–0.7	−1.1 ± 0.9	−3.7–0.7	0.38
Language	0.1 ± 0.9	−2.2–1.5	0.1 ± 0.3	−2.2–1.5	−0.7 ± 0.8	−3.7–2.1	0.65
Episodic Memory	−0.1 ± 0.8	−2.7–1.5	−0.1 ± 0.2	−1.9–1.3	−0.3 ± 0.3	−4.9–1.2	0.95
Executive Function	0.0 ± 0.5	−1.3–0.9	−0.5 ± 0.2	−1.77#x02013;0.9	−1.1 ± 0.3^a,b^	−3.5–0.3	<0.001

a: is significantly different from controls (*p* < 0.05); b: is significantly different from patients with left cerebellar infarction (*p* < 0.05). Abbreviations: SD, Standard deviation.

The lesion distributed across lobules IV to X, concentrated on lobules Crus I and Crus II, mainly on the right side (Figure 3). To evaluate the effect of lesion location on cognitive function, the lesion of each cerebellar infarction patient was divided according to a cerebellar lobule. An impaired cognitive domain was defined as one or more SD below healthy group means. According to ACE-III, patients whose lesion involved lobule VI, VIII, and IX had highest prevalence of cognitive impairment with the rate of 64.7%, 43.5%, and 40% respectively. In addition, when lobule VI was damaged, attention and working memory had the lowest *z* score (*z* attention = −1.38; *z* working memory = −0.76), and 28 (62.5%) and 29 (64.7%) patients were impaired in the cognitive domain of attention and working memory respectively. When lobule Crus I was damaged, the *z* score of executive function was lowest (*z* = −0.98). The damage lobule VIIIB and IX had the lowest *z* score for language (−0.93), while the damage lobule X and IX had the lowest *z* score for visuospatial (−0.58) and episodic memory (−0.15; Figure 4). Furthermore, the data implicated that lobule VI, VIII and IX as the prevalent areas of lesion overlap that are related to deficits in attention, working memory and executive function (Figure 5).

RETRACTED

**Figure 3:** Flattened representation of the cerebellum **(A)** and the patients’ lesion distribution in this Study **(B)**.

**Figure 4:** Hot spot figure of *z*-transformed scores of different cognitive domain, grouped according to lobular lesion topography.

**Figure 5:** Hot spot figure of the percentage of patients who were impaired in each cognitive domain, grouped according to lobular lesion topography. Description: Impaired cognitive domain was defined as *z*-score ≥ one standard deviation below healthy group means. The gray scale indicates the percentage of patients with impaired cognitive performance whose lesions involved a given lobule.

As shown in Figure 6, the global cognitive function showed a negative association with lesion volume, and the correlation coefficient was −0.37 (*p* = 0.04).

**Figure 6:** The association between global cognitive function and lesion volume in patients with cerebellar infarction.

## Discussion

In the current study, we confirmed the cognitive impairment in cerebellar infarction, which is predominant in attention and executive dysfunction. Compared with the left lesions, patients with right cerebellar hemisphere damage had worse psychological performance, suggesting cerebellar cognitive lateralization. In addition, we also found the important contributions of the cerebellar posterior lobe (especially lobules VI, VIII, and IX) to cognition.

In the current study, we applied the ACE-III scale to explore cognitive function in patients with cerebellar disorders and found that the incidence of cognitive impairment is 48.9%, which was higher than in previous studies (Kalashnikova et al., 2005; Erdal et al., 2021). The possible explanation is that the most common cognitive screening tools previously applied were the Mini-mental State Examination (MMSE) and the Montreal Cognitive Assessment scale (MoCA), which were mainly focused on detecting the dysfunction of episodic memory and were not suitable for the cerebellar disease. Because the cognitive domains that ACE-III assessed are attention, execution, language, and visuospatial ability, which cover the characteristics of CCAS, we can identify cognitive impairment in cerebellar disorders more sensitively by using this scale. A recent study also showed that the ACE III is a sensitive screening tool to detect cognitive impairments in patients with cerebellar damage (Starowicz-Filip et al., 2022). Consistent with previous studies, our study also found attention and executive function were severely impaired in patients with cerebellar infarction (Schmahmann and Sherman, 1998). The prefrontal cortex (PFC) plays a substantial role in the executive controlling function, and the presence of loops between the PFC and the cerebellum has been confirmed (D’Angelo et al., 2016). CCAS is considered to result mainly from the lesions in the cerebellar posterior lobe, and consequently, the disruption of the cerebrocerebellar circuitry (Van Overwalle and Mariën, 2016; Rastogi et al., 2017).

RETRACTED

In addition, our study found that cognitive function was mildly damaged after cerebellar infarction, and less than 20% patients suffered more than three cognitively impaired domains. “Dysmetria of thought” is proposed as a fundamental framework attempting to explain the cognitive symptoms in cerebellar disease (Schmahmann, 1998). It is hypothesized that the prefrontal discharges are regulated and modulated, rather than generated, by cerebellar structures, which explains why cognitive impairments after cerebellar infarction were mild. Unlike cerebellar neurodegenerative diseases like spinocerebellar ataxia, this study focused on cerebellar infarction, in which lesions were focal. According to the cerebellar functional topography, patients with focal cerebellar lesion may only be impaired in specific cognitive domain, which provides the explanation that only a few patients in the study had multiple cognitive domains impairment.

In the current study, patients with right cerebellar hemisphere infarction manifested poorer cognitive performance than those with left-lateralized lesions. Previous studies about cerebellar cognitive lateralization remain controversial. Some of previous studies’ findings were in accordance with ours (Shin et al., 2017; Chirino-Pérez et al., 2021). The phenomenon of crossed cerebello-cerebral diaschisis (CCD) might be the explanation: cerebral perfusion and metabolism contralateral to cerebellar lesions decreased in patients with focal cerebellar lesions (Broich et al., 1987). Furthermore, functional neuroimaging studies using Single Photon Emission Computed Tomography and Near-Infrared Spectroscopy have demonstrated that cerebral hypometabolism and hypoperfusion may contribute to cognitive dysfunction in cerebellar infarction (Baillieux et al., 2010; Saita et al., 2017; Fujii et al., 2021). However, the side of the lesion showed no significant effect on cognitive performance in other studies (Tedesco et al., 2011). The possible reason is that, as bilateral cortical activation was observed during linguistic and spatial tasks, cerebral cortex functions are not always completely lateralized (Ferrara et al., 2021).

RETRACTED

We also found that patients had worse cognitive performance when the cerebellar posterior lobe (especially lobule VI, VIII, and IX) gets damaged. Previous studies have explored the functional topography by using the voxel-lesion symptoms mapping method: damage to cerebellar lobules III–VI was associated with severe ataxia symptoms, while posterior cerebellar damage involving lobules VII and VIII was associated with cognitive deficits, confirming the anterior-sensorimotor/posterior-cognitive dichotomy in cerebellum (Burciu et al., 2014; Stoodley et al., 2016; Chirino-Pérez et al., 2021). According to the hypothesis of universal cerebellar transformation (UCT), the cerebellum has a consistent internal structure, and the heterogeneity of cerebellar connections with extracerebellar structures rather than variations in cerebellar microstructure, causes the precise localization of functions in the cerebellum (Diedrichsen et al., 2019). Using diffusion tensor imaging, Wang et al. (2019) found that abnormal alterations in the right posterior cingulate gyrus, the bilateral median cingulate and paracingulate gyri, and the right precuneus may be fundamental contributors to the cognitive impairment following cerebellar infarctions. Fan et al. (2019) discovered that in individuals with acute posterior cerebellar infarction, reduced fractional amplitude of low-frequency fluctuation in the left hippocampus and right cingulate gyrus is associated with impaired cognitive function. Those functional neuroimaging studies confirmed that the cerebellum has extensive connectivity with various cerebral areas (Liu et al., 2022).

However, patients’ global cognitive function was correlated with ataxia severity in the current study, which is inconsistent with the theory of motor-cognitive dichotomy (Schmahmann et al., 2009; Shin et al., 2017). The reason may be that larger infarcts had more impaired cerebellar lobules which caused worse performance, and patients with larger infarctions had more severe motor dysfunction which may influence cognitive assessment (Supplementary Figure 4).

This study focused on the role of the cerebellum in cognitive function. We described detailed cognitive profiles of patients with isolated cerebellar infarction by using various neuropsychological assessments and preliminarily explored the effect of cerebellar lesion location on cognitive function. However, our study has several limitations. First, the symptom of dizziness and headache occurring in acute or subacute cerebellar infarction patients may influence the cognitive assessment. Second, as emotion processing is associated with cognition, patients had more severe anxiety than healthy controls, which may lead to an overestimation of cognitive impairment incidence. Third, we only used a few scales to evaluate the cognitive domains of working memory, visuospatial, and language function, resulting in an inaccurate cognitive domain assessment. Finally, the effect of cerebellar lesion location on cognitive function was merely descriptive due to the small sample size of this research, and the motor-cognitive dichotomy pattern were not able to be validated because only four patients had infarcts in the anterior cerebellum in the current study. It should be cautious in extrapolating the data in this study, and future research with larger cohorts should be conducted.

RETRACTED

## Conclusion

This study identified that the cerebellum played a modulatory role in cognitive function, especially in attention processing and executive function. We also revealed the right-sided lateralization of cognition and functional topography in the cerebellum. Our findings enriched the understanding of cerebellar involvement in cognition. Recently, the CCAS scale has been developed as a bedside screening tool to improve the diagnosis of the CCAS in clinical contexts (Hoche et al., 2018), and more studies are needed to explore the characteristics of cognitive function in cerebellar disorders by using this scale. Furthermore, as non-invasive stimulation techniques have been applied for cognitive rehabilitation, our findings suggested that the cerebellum may be a target to improve cognitive deficits, and more research will be required in the future.

## Data Availability Statement

The original contributions presented in the study are included in the article/Supplementary material, further inquiries can be directed to the corresponding author.

## Ethics Statement

The studies involving human participants were reviewed and approved by Beijing Tiantan Hospital. The patients/participants provided their written informed consent to participate in this study.

## Author Contributions

YZ had full access to all of the data in the study, takes responsibility for the integrity of the data, and the accuracy of the data analysis. QL contributed to the study concept, performed statistical analysis, and drafted the article. CL and YZ revised the manuscript for important intellectual content. All authors contributed to the article and approved the submitted version.

## Funding

Funding for this study was provided by the National Key R&D Program of China (2018YFC2002300, 2018YFC2002302, and 2020YFC2004102) and the National Natural Science Foundation of China (81972144).

RETRACTED

## Footnotes

^1^ https://ww2.mathworks.cn

^2^ https://www.fil.ion.ucl.ac.uk/spm/software/

^3^ https://www.slicer.org
